The article "Neoadjuvant Therapy for Esophageal Adenocarcinoma in the Community Setting—Practice and Outcomes" was retracted in 2019. Reason: lack of ethics approval or compliance.

# Neoadjuvant Therapy for Esophageal Adenocarcinoma in the Community Setting—Practice and Outcomes

**DOI:** 10.3389/fonc.2017.00151

**Published:** 2017-07-18

**Authors:** Joe Abdo, Carrie A. Bertellotti, David L. Cornell, Devendra K. Agrawal, Sumeet K. Mittal

**Affiliations:** ^1^Department of Clinical and Translational Science, Creighton University School of Medicine, Omaha, NE, United States; ^2^Department of Surgery, CHI Health Creighton University Medical Center, Omaha, NE, United States; ^3^Norton Thoracic Institute, St. Joseph’s Hospital and Medical Center, Dignity Health, Phoenix, AZ, United States

**Keywords:** esophageal adenocarcinoma, molecular diagnostics, targeted therapy, proteomics, targeted chemotherapy, clinical outcomes, patient management

## Abstract

There has been an alarming rise in the incidence of esophageal adenocarcinoma which continues to have poor survival rates primarily due to lack of effective chemotherapy and presentation at advanced stages. Over a dozen chemotherapeutic agents are FDA approved for esophageal cancer (EC), and a two or three-drug combination is typically prescribed as first-line therapy for the majority of EC patients, administered either pre or post-operatively with esophageal resection. We have noticed significant variability in adjuvant and neoadjuvant regimens used in the community setting. The aim of this study was to review the various drug regimens used in the neoadjuvant setting for EC patients with adenocarcinoma undergoing resection at a single tertiary referral center in the Midwest. A total of 123 patients (stage II–III) underwent esophageal resection after neoadjuvant treatment at the center. Overall, 18 distinct drug regimens were used in 123 patients including two patients who received targeted therapy. Median survival post-surgery for this group was 11.2 months with no single regimen offering a survival advantage. These results reveal an unclear algorithm of how accepted regimens are prescribed in the community setting as well as a dire need for agents that are more effective. Additionally, it was noted that although proteomic markers have been found to predict drug response to 92% of the FDA-approved drugs in EC (12 of 13), according to pathology reports, molecular diagnostic testing was not used to direct treatment in this cohort. We therefore propose potential strategies to improve clinical outcomes including the use of a robust molecular oncology diagnostic panel and discuss the potential role for targeted chemotherapy and/or immunotherapy in the management of EC patients.

## Introduction

Esophageal adenocarcinoma (EAC) by virtue of its rapidly increasing incidence, association with gastroesophageal reflux disease and poor prognosis has received unprecedented attention in the last 15 years. There are two major types of esophageal cancer (EC): squamous-cell carcinoma which remains the most common histology worldwide, and adenocarcinoma where the prevalence is reaching an epidemic level in the western hemisphere (1). EC has some of the shortest survival durations in all of oncology. Even in 2017 a patient with a new diagnosis of EC, regardless of treatment path, can expect a median survival of 13 months (2). Stage II and III patients undergoing the present standard of care of neoadjuvant chemoradiation followed by esophagectomy surgery, have a median overall survival (OS) of just 9.0 months (3).

Surgical resection remains the backbone for treatment of loco-regional disease and outcomes for stage II and III diseases are better with adjuvant or neoadjuvant therapy (4). Surgery alone is recommended only for a small percentage of patients with early disease or those who cannot tolerate tri-modality treatment (5).

The aggressive nature of esophageal carcinoma has led to the study of combined-modality therapies incorporating chemotherapy, radiation, and surgery. More than a dozen chemotherapeutic agents are FDA approved for EC (Table 1), and a combination of two or three of these drugs are typically prescribed for first-line therapy for the majority of EC patients, either before or after surgical esophagectomy (6). Although results are available from numerous approved randomized chemotherapy trials, there is no agreement as to the best regimen for first-line chemotherapy for loco-regional or advanced EC. Chemotherapy regimens utilizing multiple agents have yielded better response rates than monotherapy. Single-drug strategies have been employed mostly for elderly EC patients due to increased toxicity and adverse drug related events for combined treatment regimens. Unfortunately, in the general EC population, even multiple chemotherapeutic agent combinations have translated to only modest improvements in OS (7). Only one-third to half of patients demonstrate a meaningful response to combined neoadjuvant regimens while 100% experience the toxic side effects (8).

**Table 1:** Precision medicine is possible in esophageal cancer (EC).

Drug	Affiliated biomarker	Brand name	Drug Status in EC	Type of treatment
Capecitabine	**TS**	Xeloda^®^	FDA approved	Chemotherapy
Fluorouracil	**TS**	Generic	FDA approved	Chemotherapy
Carboplatin	**ERCC1**	Generic	FDA approved	Chemotherapy
Cisplatin	**ERCC1**	Platinol^®^	FDA approved	Chemotherapy
Docetaxel	**TUBB3**	Taxotere^®^	FDA approved	Chemotherapy
Epirubicin	**TOPO2A**	Ellence^®^	FDA approved	Chemotherapy
Etoposide	**TOPO2A**	Etopophos^®^	FDA approved	Chemotherapy
Irinotecan	**TOPO1**	Camptosar^®^	FDA approved	Chemotherapy
Oxaliplatin	**ERCC1**	Eloxatin^®^	FDA approved	Chemotherapy
Paclitaxel	**TUBB3**	Taxol^®^	FDA approved	Chemotherapy
Mitocycin		Generic	FDA approved	Chemotherapy
Leucovorin	**RFC**	Folinic Acid	FDA approved	Chemotherapy
Trastuzumab	**HER2**	Herceptin^®^	FDA approved	Targeted therapy
Cetuximab	**EGFR**	Erbitux^®^	Off-label	Targeted therapy
Lapatinib	**HER2/EGFR**	Tykerb^®^	Off-label	Targeted therapy
Anti-PD-L1, immunotherapy	**PD-L1**	Durvalumab^®^, Atezolizumab^®^	Clinical trails	Targeted therapy

*A comprehensive list of drugs currently utilized in EC including all of the drugs prescribed to our 123-patient cohort. All of these drugs (with the exception of mitomycin) have corresponding proteomic biomarkers that act as targets for drugs or act as tumoral resistant elements if expressed. Proteomic quantification of these biomarkers could improve first-line patient management strategies in EC*.

*Green biomarker indicates improved benefit if expressed. Red biomarkers are indicative of resistance proteins and their affiliated drugs should be avoided if expressed in a solid tumor*.

*ERCC1, excision repair cross-complementation group 1; RFC, reduced folate carrier; TUBB3, tubulin beta 3; TOPO2A, type II topoisomerase; TOPO1, topoisomerase-1; TS, thymidylate synthase; HER2, receptor tyrosine-protein kinase erbB-2; EGFR, epidermal growth factor receptor; PD-L1, programmed death-ligand 1; 5-FU, fluorouracil; TKIs, tyrosine kinase inhibitors*.

Tumor reduction with neoadjuvant chemoradiotherapy is achieved in roughly half of the recipients allowing for higher R0 resection rates (9). In the preoperative therapy setting, concurrent chemoradiotherapy with 5-fluorouracil (5-FU) and cisplatin is one of the most commonly used regimens. Nonetheless, the effect of preoperative chemoradiation with 5-FU and cisplatin on survival compared to other regimens is uncertain at best. Three papers evaluating the meta-analysis of clinical trials comparing surgery alone to neoadjuvant chemoradiation and surgery demonstrated a slightly improved 3-year survival in patients with EC (5, 10, 11). However, if the Walsh et al. (12) meta-analysis is not taken into account, then there is no statistical benefit for this strategy—which currently remains the standard of care for stage II and stage III EC according to NCCN guidelines. The 5-FU, cisplatin, and radiation regimen causes severe toxicity in many patients which typically leads to hospitalization. Consequently, the best regimen of perioperative chemoradiation has not yet been established.

The use of preoperative radiation also remains controversial (13). A retrospective study looking at neoadjuvant chemoradiation vs chemotherapy alone demonstrated that the addition of radiation preoperatively yielded worse survival benefit (17 vs 21 months OS). Furthermore, the chemoradiation cohort mortality and complication rates were higher than chemotherapy alone (14). Even without proven superiority (or inferiority) of combined chemoradiotherapy vs chemotherapy alone in the neoadjuvant setting, radiation continues to be widely incorporated into EC cases (13).

The data collected over this 12 year period at our tertiary referral medical center demonstrates a wide variation in neoadjuvant treatment administered to patients with loco-regional disease prior to referral for definitive surgical resection. The aim of this study was to determine the landscape of clinical practice in the community setting for the neoadjuvant treatment of EC. We believe that this introspection calls for improved patient management strategies for this disease and a need for consistent and clear treatment plans. Furthermore, we discuss the role of targeted chemotherapy and/or immunotherapy as potential future treatment strategies for this disease.

## Materials and Methods

The Esophageal Center at Creighton University Medical Center (CUMC) is a tertiary care referral center providing surgical intervention for foregut diseases in the Midwest region. All patients undergoing surgical resection for EC at our center are entered into a prospectively maintained database that includes details of neoadjuvant treatment, operative course and long-term follow-up. After the approval of the research protocol by the Creighton University Institutional Review Board (Omaha, NE, USA), a Department of Surgery database was queried to identify patients who underwent esophageal resection between July 2004 and June 2016. Patients who underwent neoadjuvant chemotherapy or chemoradiation therapy were logged into an Excel spreadsheet. Figure 1 depicts various treatment paths a newly diagnosed patient might take, with all of the patients in our study following the perioperative protocol highlighted by the red box.

**Figure 1:** Paths to treatment in esophageal cancer (EC). Red box is the treatment path of the cohort analyzed in this study.

Only stage II and III EAC patients receiving neoadjuvant treatment (chemotherapy with or without radiation) followed by surgery were considered for this analysis. Radiation dosage for patients receiving neoadjuvant therapy is typically 4,500–5,040 cGy, split over a 4–6 week period in concert with their chemotherapy. Occasionally a slightly higher radiation dosage was used per the discretion of the treating radio oncologist.

Patients’ neoadjuvant chemotherapy regimen and radiation therapy doses were prospectively logged and retrospectively extracted. Date of surgery and date of death were used to calculate OS. Survival rates were grouped and analyzed based on regimen. We further sub-classified the regimens by drug class and correlated them with OS statistics as established by national clinical trial cooperative groups.

## Results

A total of 250 patients underwent esophageal resection between 2004 and 2016, of which 216 were for malignant disease (182 adenocarcinoma and 34 squamous-cell carcinoma). Of these, 123 patients with adenocarcinoma received neoadjuvant chemoradiation therapy at the direction of the referring oncologist(s) and this group forms the cohort for this study. First-line therapy regimens used in the 123 EAC patients are depicted in Figure 2. This pie chart reveals the broad variability of EC management strategies for patients with stage II–III disease. The chemotherapy regimens prescribed were administered by various medical oncologists in the patient’s local community. Out of 123 EAC cases, only two patients (less than 2%) had targeted therapy incorporated into their first-line regimen. Cisplatin + 5-FU was the most utilized first-line combination therapy, which was prescribed to 41 patients. The remaining 82 EAC patients received notable variation in their prescribed chemotherapy regimen and subsequent management (Figure 2).

**Figure 2:** One disease, 18 different treatments. Neoadjuvant drug regimen used in 123 patients who were referred to Creighton University Medical Center (CUMC) for esophageal resection. Pie chart affirms the variability of first-line esophageal cancer chemotherapy. Red box highlights that only 2 neoadjuvant regimen utilized targeted therapy.

Other than the two most prescribed regimens, 53% of patients were treated with one of 16 different combination chemotherapy regimens which reveals a heterogeneous distribution of patients with inconsistent first-line therapies. Approximately 30% of patients were placed on the Hopkins–Yale regimen of Cisplatin/5-FU/Radiation therapy. However, the OS for Stage IIA, IIB, III, and IV disease for patients on the Hopkins–Yale regimen was 22, 13.5, 18, and 4.9 months, respectively—which reveals an underwhelming performance for the most popular regimen of this cohort (15). However, the last EC patient referred to CUMC who was treated with this protocol was in 2012. Oncologists in our region have migrated away from the Hopkins–Yale cancer management strategy for adenocarcinoma of the esophagus.

The most widely used first-line neoadjuvant drug regimen today appears to be taxol plus carboplatin, which has been reported to have a 9- to 13-month median national survival rate (16, 17). Unfortunately, the Taxol + Carboplatin regimen performed much worse than the previous most popular regimen of Cisplatin + 5-FU in the cohort treated at CUMC (8.1 vs 12.2 months median post-operative survival). Thus, it appears from our perspective that the current most popular regimen in our Midwest region offers no greater benefit and may indeed have poorer outcomes than the former most popular regimen.

Table 2 provides a bird-eye view of the survival rates of patients treated at CUMC and sub-classified according to their neoadjuvant drug regimen. Adverse drug reactions and complication rates identified by the referring oncologist (based on the last oncology note prior to surgery) are provided by regimen. National median survival rates for these regimens are also provided. All 10 of the non-targeted regimens had neoadjuvant complications greater than 50% with some approaching a 75–100% likelihood of adverse events for these treatment selections. The median OS for the entire CUMC cohort was 11.2 months and after adjusting for the difference in start-of-therapy time points, our patient’s OS is consistent with the national statistics for stages (II–III) and course of therapy (neoadjuvant chemoradiation + esophagectomy) (3).

**Table 2:** Survival rates of patients treated at Creighton University Medical Center (CUMC) conjoined with their neoadjuvant drug regimen.

Drug class regimen utilized in cohort	Treated at CUMC (*N*)	CUMC median survival (stages II–III)	Neoadjuvant complications (CUMC cohort) (%)	Years administered (CUMC cohort)	National objective response rate (%)	National median survival (months)	Sources cohorts with no previous chemotherapy	Stage national trial cohort	Source (*N*)
Platinum + pyrimidine analog	46	12.2 months	58	2004–2012	35–41	7.7–10.5	Bleiberg et al. (18)	II–IV	92
							Cunningham et al. (19)		
Platinum + taxane	34	8.1 months	57	2012–2015	43–49	9–13	Polee et al. (16)	II–IV	86
							Zhang et al. (17)		
Platinum + taxane + pyrimidine analog	10	19.8 months	71	2006–2010	37	6.7	Ajani et al. (20)	IV	221
Platinum + topoisomerase inhibitor	9	8.7 months	75	2008–2011	48	7.0–9.8	Spirinodinis et al. (21), Kok et al. (22)	II–IV	100
ECF (Platinum + anthracycline + pyrimidine analog)	8	12.3 months	67	2008–2015	41	9.4–11.2	Cunningham et al. (23)	III–IV	1,002
FOLFOX (Folic Acid analogs + pyrimidine analog + platinum)	6	12.8 months	75	2013–2014	25–40	6.5–10.7	Warner et al. (24), Mauer et al. (25), Al-Batran et al. (26)	III–IV	285
Pyrimidine analog + folic acid analog	3	7.0 months	50	2007, 2015 (2)	29	6.8	Kok et al. (27)	IV	29
Pyrimidine analog + mitomycin	2	4.3 months	100	2007, 2010	Not available	8.0	Coia et al. (28)	I–IV	50
Pyrimidine analog monotherapy	2	3.7 months	50	2010, 2011	9	10.8	Boku et al. (29)	IV	234
Pyrimidine analog + platinum + herceptin	1	>5 years	None	2011	47	13.8	Cutsem (30) TOGA Trial	III–V	584
Pyrimidine analog + platinum + cetuximab	1	44.3 months	None	2009	57	9.4	Lordick et al. (31) EXPAND Gastric only	IV	904
Platinum monotherapy	1	N/A	N/A	2009	38	4.9	Khushalani et al. (32)	II–IV	36

Median overall survival (OS) of entire CUMC cohort—11.2 months					National median overall survival of patients treated with neoadjuvant chemoradiation and esophagectomy—9.0 months (2)				

*Complication rates for each regimen are provided. National median survival rates for these regimens are also provided. Red box highlights that the two patients who received targeted therapy in concert with chemotherapy responded well (16–32)*.

## Discussion

This report provides a view from the trenches analyzing the disarray of first-line therapy for EC patients who have been treated by community oncologists prior to referral to CUMC for definitive surgical resection. During the past 30 years, the incidence of EAC has increased dramatically, upwards of more than 400% in the Western world (33). Although progress in the therapy of local and locally advanced EACs has been made, the overall 5-year survival remains a disappointing 15–25%, with best outcomes for patients diagnosed in early stages of their disease and in concert with a favorable response to multimodal treatment (34). Unfortunately, death remains the most common outcome of EC, while the best chemotherapy regimens and the clinical utility of additive radiation remains controversial. However, the different etiologies, molecular biology, and recurrence patterns associated with malignancies of the esophagus suggest the need to identify and place patients into more concise homogeneous treatment groups rather than treating larger heterogeneous groups of EC patients with similar strategies. Clearly there exists a need to strategize beyond targeting the cell cycle *via* radiation, platins, and taxanes which are currently used in EC therapies irrespective of the varieties in genomic and proteomic expression. As it stands, the rate of EC is increasing and the arsenal to fight this disease is increasing; however, the outcomes have yet to be improved.

Eighteen different neoadjuvant regimens for 123 patients indicates a high degree of variability and unpredictability in EC therapy, further supporting that no clear regimen produces the best therapeutic response in these patients. Why has the number of therapy options increased significantly, yet survival rates remained consistently low over the last 30 years? Our findings are of a level 2a retrospective cohort of continuous prospective data, and are not the same nor nearly as significant as a randomized clinical 1a trial. Nevertheless it does reveal a different reality where patients being referred for definitive surgical resection are receiving treatment therapies prior to referral that are incongruent and inconsistent. Table 3 provides 14 other drug regimens that are either in use or under investigation for EC in the United States. This brings the total of neoadjuvant therapy options to approximately 32 combination or monotherapy choices. Some of these clinical trial drug regimens had a much better performance than the two most common drug combinations for EC. For instance, S-1 plus cisplatin demonstrated a 53% response rate and had a 13-month median survival. Irinotecan plus 5-FU plus cetuximab had a 16.6-month median OS—which is impressive yet still not ideal (35, 36). Perhaps because of EC’s aggressive nature, the oncology field has desperately developed an “everything but the kitchen sink” approach to treating this disease, utilizing platinums, taxanes, anthracyclines, topoisomerase I inhibitors or pyrimidine analogs as first-line therapy. Although our cohort received a wide-range of combination therapies, the median OS for the entire group was 11.3 months—approximately 2 months longer than the national median OS for patients with similar stages treated with similar perioperative protocols (3). We have not seen a shift in the positive direction in regards to improved response rates which could be due to a switch of histologic subtype presentation from squamous cell to adenocarcinoma in the US coinciding with the same therapeutic strategies utilized over the decades.

**Table 3:** Missed opportunities?

Other drug regimen utilized in esophageal cancer (EC)	Treated at CUMC (*N*)	Objective response rate (%)	Median survival (overall survival) (months)	Source	Clinical trial (*N*)
FOLFIRI (5-FU plus leucovorin and irinotecan)	0	39	9.5	Guimbaud et al. (37)	416
Anthracycline + taxane	0	27	8.6	Hecht et al. (38)	28
Irinotecan + 5FU + cetuximab (anti-EFGR)	0	44–46	16.6	Moehler et al. (36)	49
Cisplatin + irinotecan	0	38	12.3	Boku et al. (29)	704
Lapatinib (targets HER2 + EGFR) + chemotherapy	0	53	12.2	Hecht et al. (39)	545
Ramucirumab (targets VEGF) + FOLFOX	0	46	11.7	Yoon et al. (40)	168
Ramucirumab (targets VEGF) monotherapy	0	3	5.2	Fuchs et al. (41)	238
S-1 plus cisplatin	0	54	13	Koizumi et al. (35)	148
FAM (5-FU, doxorubicin, and mitomycin)	0	42	5.5	MacDonald et al. (42)	62
Taxane + platinum + anthracycline	0	70	10.0	Sharma et al. (43)	33
Immunotherapy (PD-1 check point inhibitor)	0	Not available	16.7	Moehler et al. (44)	57
MCF (mitomycin, cisplatin, and 5-FU)	0	44	8.7	Ross et al. (45)	580
5-FU + leucovorin (LV5FU2)	0	13	6.8	Bouché et al. (46)	136
5-FU + mitomycin + leucovorin	0	39	11.3	Kim et al. (47)	48

*Other FDA-approved drug regimen for EC that were not utilized by the Midwestern community oncologists who referred their patients to Creighton University Medical Center (CUMC) for esophagectomy. A number of these regimen performed much better in national clinical trials than many of the preferred regimen used in our cohort (29, 35–47)*.

Finally, only two patients (<2%) of the 123 patients received targeted therapy. In this era of molecular oncology, it is disconcerting that such a small proportion of patients received targeted therapy which has been associated with improved outcomes in a myriad of solid tumor indications. HER2 is overexpressed in 20–33% of EAC tumors, and EGFR is overexpressed in 25–30% of gastroesophageal tumors—demonstrating missed opportunities to potentially improve outcomes utilizing targeted therapies in our cohort (48, 49). Eight clinical trials testing EGFR targeted therapy with tyrosine kinase inhibitors (TKIs) vs chemotherapy in first-line non-small cell lung carcinoma demonstrated significant improvements in response rates and OS for every cohort treated with targeted therapy (50). Some of these trials had double or triple progression-free survival rates for patients who received targeted therapy in the first-line setting compared to patients who received only chemotherapy (50). The ToGA trial also demonstrated an improved response rate and survival outcomes utilizing HER2 targeted therapy in gastroesophageal cancers (51). In this trial patients received HER2 targeted therapy irrespective of HER2 expression status, thus the response and survival rates could have been further improved had the cohorts been preselected based on the target actually represented in the tumor. The two patients in our cohort who received neoadjuvant targeted therapy did have longer survival compared to the other groups, but given this small sample size, meaningful conclusions cannot be drawn from our study.

### Limitations

Our study only takes into account patients in a single center in the Midwest representing a small cohort retrospective review of our prospective data. The environmental factors and patient population were largely homogeneous, comprised of mostly white males in their 60s, which is representative of the national demographics for EAC. We also calculated OS from the time of surgery, rather than from the day neoadjuvant therapy was instituted. Therefore, these data points may be 4–12 weeks shorter than their actual survival time. This paper also focused on patients who were Stage II and III. There could potentially be more adherence to oncology guidelines in the stage I or metastatic settings. The lack of targeted therapy used in these 123 patients has been noted. Is it possible that pathological services and outsourced diagnostics or insurance coverage for our cohort are not entirely available to some of our patients and/or oncologists—concealing information or preventing optimal first-line therapy in these patients? It is also conceivable that some patients may have received targeted therapy in the (post-operative) adjuvant setting.

### How to Improve

When most people hear of companion diagnostics and personalized medicine, they think of assays that are exclusively affiliated with targeted therapies. However, there is now accumulating evidence that shows how proteomics can also be used to personalize chemotherapy regimens (52, 53). Specifically, three proteins [excision repair cross-complementation group 1 (ERCC1), TUBB3, thymidine synthase (TS)] have been linked to decreased tumor response *via* chemoresistance. Three additional proteins [reduced folate carrier protein (RFC), TOPO1, TOPO2A] have been identified as effective targets for specific chemotherapies that have demonstrated improved therapeutic responses in other solid tumors. Furthermore, three targeted therapy markers (HER2, EGFR, PD-L1) have validated clinical utility in the patient management strategies for EC. The presence of HER2 and EGFR markers can help physicians identify patients who may be potential candidates for therapies targeting extracellular growth factors which can disrupt cellular proliferation. Whereas, tumoral PD-L1 expression can identify patients who potentially may have a favorable response to a number of immune checkpoint inhibitors. Herein, we propose a 9-marker panel which has been identified as being predictive of improved or decreased tumor responses with the drugs that are FDA approved for EC (Table 1). The expression status of these 9 proteins are associated with 92% of the approved drugs in EC, can be determined *via* multiplexed immunohistochemistry or mass spectrophotometric analysis, and could assist in optimizing first-line therapy in EC (Figure 3). Six of these markers (HER2, EGFR, PD-L1, TS, ERCC1, and TUBB3) have proven clinical utility specifically in EC patients. The remaining three markers (RFC, TOPO1, and TOPO2A) have not been specifically validated in esophageal cohorts but based on basic biochemical interactions may be efficacious in predicting a tumor’s response to specific classes of drugs.

**Figure 3:** A plea for sanity. Suggested proteomic expression assay panel which could assist in optimizing a first-line therapy for esophageal cancer patients. Unadulterated tumor specimen is crucial for reliable proteomic expression results which can ultimately assist in more robust precision medicine. Please consult with a pathologist on the best ways to achieve expression results on these markers. ERCC1, excision repair cross-complementation group 1; RFC, reduced folate carrier; TUBB3, tubulin beta 3; TOPO2A, type II topoisomerase; TOPO1, topoisomerase-1; TS, thymidylate synthase; HER2, receptor tyrosine-protein kinase erbB-2; EGFR, epidermal growth factor receptor; PD-L1, programmed death-ligand 1; 5-FU, fluorouracil; TKIs, tyrosine kinase inhibitors.

#### Markers with Proven Predictive Efficacy for EC Chemotherapy

Excision repair cross-complementation group 1 or ERCC1 is a protein involved in the main DNA repair system and has been associated with resistance to platinum-based therapies in a number of cancers (54, 55). This protein can recognize and excise a wide scope of DNA damage, including damage resulting from the cross-linking of platinum-based anti-cancer drugs (56). Presumably, if a tumor expresses ERCC1, it will be able to repair the destruction caused by platinum chemotherapy while sustaining cellular proliferation, and therefore the effect of platins will be marginalized *via* ERCC1 expression. A clear linkage between high expression levels of ERCC1 and decreased patient response to the platinum-based therapy has been shown (57). Patients who had tumors with high levels of ERCC1 experienced significantly shorter OS (11.1 months) compared to patients with no or low ERCC1 (33.7 months) when treated with platinum-based regimens (57). Therefore, it would be safe to say that platins should be avoided if ERCC1 is expressed in the tumor. Additionally, EAC patients with ERCC1-negative status have a significantly higher rate of complete pathological response in the first-line setting (*P* < 0.001) (58). ERCC1-negative EC patients were additionally reported to have longer OS and longer progression-free survival than patients who expressed this protein (58). ERCC1-positive status in esophageal tumors puts patients at twice the risk of cancer recurrence, irrespective of the first-line regimen (59). Markedly, 117 out of 123 patients in our cohort received a platinum-based drug in the first-line setting while studies suggest that ERCC1 is expressed in 40% of esophageal tumors, placing a significant number of patients at risk of therapeutic inefficacy and preventable physiologic toxicity (58).

Tubulin beta 3 or TUBB3 is an intracellular marker that is associated with resistance to taxane-based therapies (60, 61). Taxanes are a drug class that acts by stabilizing microtubules, thereby preventing mitosis in rapidly proliferating cells. The main function of TUBB3 is the destabilization of microtubules, thereby allowing cellular proliferation to proceed uninhibited. It is because of this relationship that high expression of TUBB3 has been shown to inhibit taxane-based therapies in a number of cancers. In gastric tumors, high TUBB3 expression had a significantly lower response rate (16.7%) to docetaxel then tumors with low TUBB3 expression (64.3%) (62). Another study which quantified TUBB3 *via* mass spectrometry, compared gastroesophageal cancer patients with high or low TUBB3 expression in a cohort treated with taxanes (63). Patients with low TUBB3 (<700 amol/µg) had nearly double the survival duration (1,566 days) compared to patients with high expression of TUBB3 (801 days) (63). Another study reported TUBB3 expression as a predictor of response to taxanes for recurrent and metastatic gastrointestinal carcinoma (64). They demonstrated that patients with metastatic disease who had low TUBB3 expression had double the survival length (6.7 vs 3.6 months) when treated with taxanes (64).

Thymidine Synthase is a well-described enzymatic protein which acts as a resistance marker against 5-FU and capecitabine (65). 5-FU and capecitabine are pyrimidine analogs that work by inhibiting nucleoside metabolism by incorporating itself into RNA and DNA with synthetic uracil or thymine nucleobases, leading to cytotoxicity and apoptosis (66). TS works against these mechanisms by catalyzing the production of thymidylate, which plays a role in upregulating protein synthesis while avoiding programmed cell death (66). EC patients who were treated with capecitabine had double the OS duration when their tumors expressed low TS scores compared to EC patients with high TS levels (57). Another study measuring protein expression *via* surrogate mRNA levels reported that gastroEAC patients with low TS expression levels had an OS of 43 months with 5-FU based regimens. Whereas patients with TS expression above the median cutoff had an OS of just 6 months, confirming substantial resistance to 5-FU (67). Prognostically, the presence of TS in esophageal tumors was found to have a twofold greater chance of cancer recurrence, regardless of the first-line regimen (59). 79 out of 123 patients in our cohort (64%) were placed on a pyrimidine analog in the first-line setting while 35% of EC patients are positive for TS expression (58).

#### Markers with Proven Predictive Efficacy to EC Targeted Therapy

An important conclusion of this study is the lack of targeted therapies utilized in this cohort undergoing surgery at CUMC. Therefore, our call to action would be for an increased use of targeted therapies in concert with tailored chemotherapies with an increased interest in utilizing immunotherapy. High HER2 and EGFR expression are associated with improved responses to trastuzumab and TKIs, respectively (68–73). Tumoral PD-L1 expression has also been associated with improved response to a number of immunotherapies targeting various immune system-affiliated ligands (74, 75). The clinical utility of proteomics-guided therapy has already been elucidated in previous studies using EC patient samples. The increased benefit of antibody-based therapies targeting tumors with high expression of HER2, EGFR, or PD-L1 has been well described in many cancers, including EC (71, 76–78).

#### Markers with Potential Efficacy Predicting Response to EC Chemotherapy

There are three intracellular biomarkers which have not been specifically studied in EC cohorts, yet their expression levels have been associated with improved benefit in a number of solid tumor cancers. Expression of RFC has demonstrated improved response to leucovorin (79). RFC acts like a transcellular ferry by which folates are delivered into cells from the systemic circulation, and RFC-mediated transport of folinic acid (leucovorin) has been well described (80). Drugs like leucovorin, which are classified as anti-folates, can sneak into cancerous cells thru the RFC “door” and disrupt DNA synthesis thereby halting cellular proliferation (81). Greater RFC expression likely increases leucovorin’s access into malignant cells. Leucovorin has the strongest affinity to RFC protein of all the anti-folates, significantly higher than methotrexate and pemetrexed (82). Without RFC expression, the essential effects of resistance can be expected when administering leucovorin (83).

Type I topoisomerase (TOPO1) is an enzyme that, when highly expressed in a tumor, is associated with improved response to topoisomerase inhibitors such as irinotecan (84). The TOPO1 protein is affixed to DNA, induces a double stranded break, relaxes coils, and then reanneals the break. Drug molecules like irinotecan attaches to TOPO1 forming a complex that slides down DNA impairing TOPO1’s ability to reanneal the DNA break, and thereby causing premature apoptosis (84). Although the diagnostic value of TOPO1 has not been analyzed specifically in EC, it has been shown that if TOPO1 is not active in tumor cells, then drugs like irinotecan will have little to no effect in preventing proliferation and will most likely induce adverse effects in other organs of the body. TOPO1 is highly expressed in 55.2% of EC patient tumors while only 7% of our cohort received a topoisomerase inhibitor, highlighting many missed opportunities to inhibit a tumor’s ability to repair its DNA (85).

Biomarker topoisomerase 2α (TOPO2A) is affiliated with improved response to anthracyclines such as epirubicin and doxorubicin (86). TOPO2A controls and alters the topologic states of genetic code as it condenses, separates, and relieves torsional stress during the transcription and replication of DNA (87). Anthracyclines have an affinity to the TOPO2A protein and when forming a complex can inactivate the replication process that arrests cellular proliferation. TOPO2A is expressed in 48.7% of EC tumors with 24.14% of EC tumors being pathologically considered overexpressed (88). TOPO2A has also been deemed a prognostic factor in EC patients as tumors with no TOPO2A expression survived almost a year longer than patients with low to high TOPO2A expression (89). Also, TOPO2A expression in esophageal tumors has been associated with worse cellular differentiation and more perineural invasion—illuminating a potentially greater role for anthracyclines in suppressing the aggressiveness of TOPO2A positive tumors (89).

While RFC, TOPO1 and TOPO2A have not been specifically validated in EC patients, based on biochemical mechanisms of action, it would be valuable to consider multiplexed molecular diagnostics to identify the status of these tumor targets along with the three validated resistance markers (ERCC1, TUBB3, TS) and the three antibody-based therapy targets (HER2, EGFR, PD-L1) in an effort to augment first-line therapy choices (Figure 4).

**Figure 4:** Clinical utility of 9-marker panel: expression matters. Proteomic biomarkers affiliated with improved response to targeted or chemo therapy as well as resistance to various approved chemotherapeutic agents. Knowing the expression status of these biomarkers could improve patient management strategies in esophageal cancer (EC). **(A)** *Markers with potential efficacy predicting response to EC chemotherapy*. The left frame demonstrates how high expression of TOPO1 can be effective for topoisomerase inhibitors like irinotecan by forming a complex and disrupting DNA synthesis. TOPO2A and anthracyclines react in a similar way where they form a complex to inactivate DNA synthesis. Both of these mechanisms are dependent upon the formation of a complex resulting in reduced cellular proliferation and an increase in tumor regression. RFC acts like a ferry for the anti-folate drug leucovorin and is dependent on RFC to cross into the cytoplasm of a tumor cell. Once inside the cells, the leucovorin can work as an anti-folate and inhibit cellular proliferation. Greater RFC expression likely increases leucovorin’s access into malignant cells. The right side of the frame demonstrates how low expression of these markers would produce low patient response when treated with these types of drugs. **(B)** *Markers with proven predictive efficacy to EC targeted therapy*. When HER2 and EGFR is expressed in a tumor they can be utilized to inhibit cellular growth *via* targeted therapy. Blocking these proteins with monoclonal antibodies prevents their ability to send growth factor signals which results in tumor regression. Blocking the PD-L1 ligand expressed on a tumor allows for antigen presenting cells (APCs) to come in contact with the tumor uninhibited which causes the activation and infiltration of T-cells directed at the tumor resulting in tumor regression. **(C)** *Markers with proven predictive efficacy for EC chemotherapy*. When markers ERCC1, TUBB3 and TS are expressed they act as resistance elements to platinums, taxanes and pyrimidine analogs, respectively. When these markers are not expressed, these classes of drugs can act on tumor cells uninhibited which results in increased tumor regression. The effects of these resistance markers have been tested and validated specifically in EC. ERCC1 excision repair cross-complementation group 1; RFC, reduced folate carrier; TUBB3, tubulin beta 3; TOPO2A, type II topoisomerase; TOPO1, topoisomerase-1; TS, thymidylate synthase; HER2, receptor tyrosine-protein kinase erbB-2; EGFR, epidermal growth factor receptor; PD-L1, programmed death-ligand 1.

### A Plea for Sanity

The cadre of drug treatment protocols available to treat EAC is quite large; however, there is little direction or clarity on how to implement the best regimen (Table 1). In our 123 patient cohort, 18 different drug regimens were used in the neoadjuvant setting and results are underwhelming. Less than two percent of our cohort received targeted therapy concomitantly with a platin and 5-FU. There are more than 32 treatment regimens an oncologist can choose to implement for their patient with EC (Tables 2 and 3). How can pathologists or the molecular diagnostics industry help an oncologist decide which of the 32 drug regimens is the optimal choice? An increased utilization of molecular diagnostics could help direct oncologists toward which avenue to pursue when treating this disease. In order to scrutinize the proteomic milieu of these tumors prior to chemotherapy, which disrupts the biochemical profile of the cancer, it would be helpful to attain ample formalin-fixed paraffin embedded tissue of the tumor *via* endoscopic biopsies. If patients first undergo esophageal resection before adjuvant chemoradiation, then there will be plenty of unadulterated tumor tissue to perform proteomic diagnostics for our suggested 9-marker panel (Figure 3). This would allow pathologists or molecular diagnostic companies the ability to analyze the tumor for expression of relevant proteins that have been affiliated with improved response or therapy resistance (Figure 4). Since the management of EC is so unsettled, and survival rates have remained poor, the increased utilization of targeted therapies (including immunotherapy) in concert with clinically relevant diagnostic panels would bring clarity in treating these patients and could potentially enhance survival outcomes.

We believe there is ample evidence to support routine use of the proposed 9-marker panel for improved management of patients with EAC. This includes three markers of resistance to platinums, taxanes and pyrimidine analogs (ERCC1, TUBB3, TS) which have been validated in EC cohorts. Three markers that predict response to targeted therapies (HER2, EGFR, PD-L1) have also been validated in EC patient studies. And three markers that may predict improved response to leucovorin, topoisomerase inhibitors and anthracyclines (RFC, TOPO1, TOPO2A) in EC. Insights gained from such a panel would not only guide the use of more effective regimens but also help physicians avoid non-beneficial and potentially harmful agents. This panel can be implemented and achieved with pathology-based proteomics, using either inter-hospital pathology departments or outsourced diagnostic companies, and could help optimize first-line patient management strategies. Please consult with a pathologist on the best ways to attain expression data for these markers. Our results feature regressing survival statistics, unpredictable regimen prescription, excessive therapeutic choices, and elevated adverse event rates which prompted our petition to implement enhanced precision medicine for EC cases.

## Author Contributions

JA wrote the original draft, performed survival statistics, and physically created the figures. CB provided and interpreted the de-identified patient data, tracked down supplementary data points and offered clinical expertise in the revisions. DC adjusted the language to be more accurate in terms of EC management in the clinic as well as provided two major revisions. DA supported this research with his R01 grants as well as formulated the hypothesis, provided numerous revisions, and designed a number of figures. SM brought these clinical issues to the attention of our group, he released this de-identified data of his patients to us, provided multiple drafts, adjusted figures, and with JA and DA, devised ways to potentially improve EC patient care post-esophagectomy.

## Conflict of Interest Statement

The authors have no other relevant affiliations or financial involvement with any organization or entity with financial interest or financial conflict with the subject matter or materials discussed in the manuscript apart from those disclosed. No writing assistance was utilized in the production of this manuscript.
